The article "COVID-19 in Iran: Forecasting Pandemic Using Deep Learning" was published in 2021. Journal: Comput Math Methods Med.

# COVID-19 in Iran: Forecasting Pandemic Using Deep Learning

**DOI:** 10.1155/2021/6927985

**Published:** 2021-02-25

**Authors:** Rahele Kafieh, Roya Arian, Narges Saeedizadeh, Zahra Amini, Nasim Dadashi Serej, Shervin Minaee, Sunil Kumar Yadav, Atefeh Vaezi, Nima Rezaei, Shaghayegh Haghjooy Javanmard

**Affiliations:** ^1^Medical Image and Signal Processing Research Center, School of Advanced Technologies in Medicine, Isfahan University of Medical Sciences, Isfahan, Iran; ^2^Snap Inc., Machine Learning Research Team, Seattle, WA, USA; ^3^Nocturne GmbH, Berlin, Germany; ^4^Department of Community and Family Medicine, School of Medicine, Isfahan University of Medical Sciences, Isfahan, Iran; ^5^Department of Immunology, School of Medicine, Tehran University of Medical Sciences, Tehran, Iran; ^6^Applied Physiology Research Center, Isfahan Cardiovascular Research Institute, Isfahan University of Medical Sciences, Isfahan, Iran

## Abstract

COVID-19 has led to a pandemic, affecting almost all countries in a few months. In this work, we applied selected deep learning models including multilayer perceptron, random forest, and different versions of long short-term memory (LSTM), using three data sources to train the models, including COVID-19 occurrences, basic information like coded country names, and detailed information like population, and area of different countries. *The main goal is to forecast the outbreak in nine countries (Iran, Germany, Italy, Japan, Korea, Switzerland, Spain, China, and the USA).* The performances of the models are measured using four metrics, including mean average percentage error (MAPE), root mean square error (RMSE), normalized RMSE (NRMSE), and *R*^2^. The best performance was found for a modified version of LSTM, called M-LSTM (winner model), to forecast the future trajectory of the pandemic in the mentioned countries. For this purpose, we collected the data from January 22 till July 30, 2020, for training, and from 1 August 2020 to 31 August 2020, for the testing phase. Through experimental results, the winner model achieved reasonably accurate predictions (MAPE, RMSE, NRMSE, and *R*^2^ are 0.509, 458.12, 0.001624, and 0.99997, respectively). Furthermore, we stopped the training of the model on some dates related to main country actions to investigate the effect of country actions on predictions by the model.

## 1. Introduction

An outbreak of pneumonia with an unknown origin was reported in Wuhan, China, last December 2019 [1]. The World Health Organization named this disease COVID-19 after its genetic sequencing revealed the same origin of the etiologic agent with corona viruses [2–4]. From the beginning of the epidemic till 22 Oct. 2020, more than 41,000,000 confirmed cases and more than one million deaths had been reported [5].

One of the most important concerns in dealing with influenza-like illness (ILI) pandemics such as COVID-19 is early identification and short-term estimation of its final size and peak time. This early prediction using mathematical and statistical models and combining with existing data would effectively help the governments and public health officials put in place appropriate prevention and control strategies [6, 7]. For answering this issue, many mathematical models are already used for predicting ILI pandemics. Fang et al. [8] investigated the effect of early recommended or mandatory measures on reducing the crowd infection percentage, using a crowd flow model. Roosa et al. [9] used phenomenological models that have been validated during previous outbreaks to generate and assess short-term forecasts of COVID-19. Kucharski et al. [10] combined a mathematical model of severe SARS-CoV-2 transmission with four datasets. Peng and colleagues [11] analyzed the COVID-19 epidemic in China using dynamical modeling to estimate the key epidemic. A. Remuzzi and G. Remuzzi [12] analyzed the COVID-19 situation in Italy and found its similarity to China. Sajadi et al. [13] tried to predict potential spread and seasonality for COVID-19 based on temperature, humidity, and latitude information. Mangoni and Pistilli [14] suggested a dynamical model, a developed generalized SEIR model based on [11], to make predictions on the COVID-19 outbreak using the Italian Dipartimento della Protezione Civile data. Anastassopoulou et al. [15] estimated the main epidemiological parameters, particularly the case fatality and case recovery ratios based on a susceptible-infectious-recovered-dead (SIRD) model with 90% confidence intervals. They adopted an autoregressive integrated moving average (ARIMA) model on the data collected from 31st January 2020 to 25th March 2020 and verified it using the data collected from 26th March 2020 to 04th April 2020. Khan and Gupta [16] proposed an autoregressive integrated moving average (ARIMA) model to predict the number of COVID-19-infected cases in India.

Based on some prominent studies in this field [17, 18], software computing methods, especially deep learning methods, conquered other classical models in the short-term estimation of pandemics. Given the novelty of the COVID-19 research, most studies have already focused on short-term prediction, and a limited number of works are already published on prediction and diagnosis of COVID-19 using deep learning models [19]. Ayyoubzadeh et al. [20] used a linear regression model and LSTM to predict the incidence of COVID-19 using Google trends on daily incidence data achieved from the Worldometer website from 15 February to 18 March 2020 in Iran. Zeroual et al. [21] presented a comparison of five deep learning methods, simple recurrent neural network (RNN), long short-term memory (LSTM), bidirectional LSTM (BiLSTM), gated recurrent units (GRUs), and variational autoencoder (VAE) algorithms, to predict the number of new cases and recovered cases. Chimmula and Zhang [22] aimed to forecast the future COVID-19 cases and the possible end of the outbreak in Canada using a long short-term memory (LSTM) network. Chatterjee et al. [23] applied different univariate “long short-term memory (LSTM)” models to forecast COVID-19 new cases and deaths. They concluded that vanilla, stacked, and bidirectional LSTM models outperformed multilayer LSTM models. Wieczorek et al. [24] suggested a neural network model for predicting the COVID-19 outbreak and reported accuracy above 99% in some. Melin et al. [25] used a multiple ensemble neural network model with fuzzy response aggregation to predict time series of the COVID-19 in Mexico. Liu et al. [26] investigated three different models, a modified susceptible-exposed-infected-recovered-dead (SEIRD), a long short-term memory (LSTM), and a geographically weighted regression (GWR), for prediction of the spread of COVID-19 cases in China. They reported all three models performed well, comparing their accuracy. Gao et al. [27] developed an ensemble model using four machine learning methods, logistic regression, support vector machine, gradient boosted decision tree, and neural network, to predict mortality risk of COVID-19 using clinical data of patients.

This study provides a deep learning-based prediction method that can assist medical and governmental institutions in preparing and adjusting as pandemics unfold. To this end, we utilized multiple models describing the epidemic and compare their performances and effective features in forecasting. To make sure our methodology is generalizable, in addition to data of Iran (which is our main focus in this paper), we also apply this framework to several other countries and show consistent findings for all of them. Finally, we select the winner model and compare its predictions with the real data. We show that country actions may change the predicted trend and cause a deviation between prediction and real data.

The structure of the rest of this paper is as follows.  Section 2.1 presents the details of the data sources used in this study.  Section 2.2 gives a quick introduction to the machine learning algorithms used for training a predictive model.  Section 3 provides a detailed quantitative and qualitative analysis of forecasting accuracy in Iran and other countries. Furthermore, the method investigates the effect of government policy on the number of infected cases. Finally, the paper is concluded in Section 4 by discussing the current situation and the future of COVID-19 in Iran based on the current data.

## 2. Materials and Methods

### 2.1. Research Data

This study uses three data sources to predict COVID-19 disease, including COVID-19 data, basic information, and detailed information for each country. The COVID-19 data (by John Hopkins University) contains the daily number of confirmed/death/recovered people [28] .The basic information contains information about the date/country/province of the cases. The detailed information for each country (according to information in [29]) includes information such as region/population/area (sq. mi.)/pop. density (per sq. mi.)/coastline (coast/area ratio)/net migration/infant mortality (per 1000 births)/GDP/literacy (%)/climate/birthrate/death rate/agriculture/industry/service/arable (%)/crops (%). Data of all countries provided by John Hopkins University from January 22 till July 30, 2020, were used as the training set. The training data is further divided into train and validation subsets using a ratio of 7 : 3 based on the dates. The performance in the test stage was evaluated based on the data between 1 August 2020 and 31 August 2020 from nine countries (Iran, Germany, Italy, Japan, Korea, Switzerland, Spain, China, and the USA). We predict the upcoming days from 31 August 2020 to provide forecasting on the number of confirmed, deaths, and recovered in all nine countries.

### 2.2. Analysis Method

In the proposed method, first, the relevant information is extracted and processed from data sources. Those models are then trained on COVID-19 data. Finally, the performances of the models are measured using the mean average percentage error (MAPE), root mean square error (RMSE), NRMSE, and *R*^2^ metrics. We experimented with different machine learning models and reported the result of five promising ones, which includes random forest (RF) [30], multilayer perceptron (MLP) [31], long short-term memory (LSTM) [32] with regular features (LSTM-R), LSTM with extended features (LSTM-E), and multivariate LSTM (M-LSTM). Different structures (hyperparameters and parameters) are examined for each of these models, and the best performing architectures are summarized in Table 1. As shown in Table 2, features of each country (such as basic and detailed features and lag (previous occurrences) explained in Section 3.1) are utilized as input parameters. For comparison of the models, MAPE, *R*^2^, RMSE, and NRMSE parameters are calculated as the performance metric. Each model is applied to the data separately. We used implementation in the Keras package in the Python version 3.7.3 [33].

For comparing different models, MAPE in percentage terms, RMSE, NRMSE, and *R*^2^ metrics are used to measure the size of the error regarding the actual values. These metrics are calculated using Equations (1)–(6):

(1) $$\begin{array}{c} \text{MAPE}=\frac{100}{n}\overset{n}{\underset{t=1}{\sum }}\left\|\frac{X_{t}-Y_{t}}{X_{t}}\right\|, \end{array}$$

(2) $$\begin{array}{c} \text{RMSE}=\sqrt{\frac{1}{n}\overset{n}{\underset{t=1}{\sum }}{\left(X_{t}-Y_{t}\right)}^{2}}, \end{array}$$

(3) $$\begin{array}{c} R^{2}=1-\frac{{\text{SS}}_{\text{res}}}{{\text{SS}}_{\text{tot}}}, \end{array}$$

(4) $$\begin{array}{c} {\text{SS}}_{\text{tot}}=\overset{n}{\underset{i=1}{\sum }}{\left(X_{t}-\bar{X}\right)}^{2}, \end{array}$$

(5) $$\begin{array}{c} {\text{SS}}_{\text{res}}=\overset{n}{\underset{i=1}{\sum }}{\left(X_{t}-Y_{t}\right)}^{2}. \end{array}$$

In an ideal condition, the observed values and predicted values are identical (*R*^2^ = 1). On the other hand, if *R*^2^ = 0.5, almost half of the observed variation can be explained by inputs of the model. The normalized root mean square error (NRMSE) is also used to compare models with different scales. This factor is the fraction RMSE on the observed range of data:

(6) $$\begin{array}{c} \text{NRMSE}=\frac{\text{RMSE}}{X_{\max}-X_{\min}}, \end{array}$$

where *X*_*t*_ is the actual value, *Y*_*t*_ is the corresponding estimated value for the *t*^th^ sample, *X*_max_ is the maximum, *X*_min_ is the minimum value, and $\bar{X}$ is the average of actual values from all *n* available samples.

#### 2.2.1. Random Forest

One of the models used in our work is random forest (RF) [27]. RF is essentially an ensemble of decision trees; it predicts the target value by training several decision trees and combining their results. One nice feature of RF is that it can be used for both regression and classification problems. Once the model is trained, the average predicted score of different trees can be used to predict the value of test samples. The two most popular ensemble methods are bagging and boosting. In bagging, individual models are trained in parallel by a random subset of the data [30].  Figure 1 shows the overall diagram of a RF. RF is a bagging method and parallel trees work in random forests without any interaction among them (Tree 1, Tree 2,…, Tree *M* in Figure 1). A random sample is selected repeatedly from the training set, and with the different replacement of the training set, the trees fit these samples. During the training time, all parallel trees work, and the mean prediction of the individual trees (Average *C*_*i*_) is reported as an output of RF.

#### 2.2.2. Multilayer Perceptron (MLP)

Multilayer perceptron (MLP) is a popular neural network, which uses a cascade of several nonlinear transformations to make a prediction. In this network, there are at least three layers of nodes, the input features are sometimes called the input layer, and the intermediate transformations are called the hidden layer. The outputs of the first layer (input) are used as the inputs of the next layer (hidden); this continues until, after a certain number of layers, the output of the last hidden layer is used as the input of the output layer. All nodes in hidden layers use a nonlinear activation function.

The output in the last layer is called the predicted output. In all supervised learning algorithms, the actual output is called the expected output. Expected outputs are used to measure the performance of the neural network system. Based on the expected output and predicted output values, the amount of loss of the MLP network is calculated. The calculated loss amount is used to propagate the error in the MLP and update the weights.

After calculating the amount of loss in the previous step, this value is propagated from the output layer to the first layer in the network, and using the concept of a gradient, the weights of the multilayer perceptron neural network are updated. In Figure 2, the structure of the MLP network was shown. In this study, we have used a model with 5 hidden layers. The detailed information about all layers is explained in Table 1.

#### 2.2.3. Long Short-Term Memory (LSTM)

LSTM is an artificial recurrent neural network (RNN) architecture in deep learning. Unlike standard feedforward neural networks, LSTM contains feedback links [29]. Time series adds the complexity of a sequence dependency among the input variables [32] and ideally requires a model with the sequential processing capability. The vanilla neural networks (such as MLP) do not have sequential processing power. However, there is an extension of feedforward neural networks for this purpose, called recurrent neural networks, where at each step, the input from the current time and the hidden state from the previous timestamp is used to make a prediction.  Figure 3 illustrates the overall structure of the LSTM model. In this study, we have used a model with two LSTM and two dense layers with 64, 32, 32, and 1 filters (nodes) in each layer. This information is listed in Table 1.

*(1) LSTM with Regular Features (LSTM-R)*. In this application of LSTM, we originally deal with three different occurrences: the number of confirmed/death/recovered people. Using regular features, we feed lagged samples of each occurrence to predict the next values (a single-input and single-output (SISO) format).

*(2) LSTM with Extended Features (LSTM-E)*. By adding extended occurrences from the other two types to predict the next value for each class (confirmed/death/recovered), we accept a multi-input and single-output (MISO) format.

*(3) Multivariate LSTM (M-LSTM)*. An alternate time series problem is the case where there are multiple parallel time series and a value must be predicted for each. Now, we may consider the number of occurrences in all classes (confirmed/death/recovered) as input data and predict the value for each of the three time series for the next time step (a multi-input and multioutput (MIMO) format).

## 3. Results

The machine learning models are trained and tested based on 84,372 occurrences of the daily number of confirmed, death, and recovered COVID-19 cases. A lag of six days was applied to the data. The dataset is divided into training and test data sets. Each model is tested with very different architectures, and the best performance is achieved with the architectures described in Table 1.

The performance of each model is evaluated on the test set with evaluation based on the MAPE, RMSE, NRMSE, and *R*^2^ values. The best lag is found by comparing MAPE values as discussed in Section 3.1. The results also changed by feeding different input features to each candidate model (elaborated in Table 1) in Section 3.2. The best model/input combinations are then found to forecast the next days in Section 3.3. The effect of country actions on predictions is also investigated in Section 3.4.

### 3.1. Optimal Lag Parameter

Assuming that we want to predict the occurrences after a time point, it is not enough to only consider the information from one single day; one needs to use information from some passing days (lag parameter). Different time intervals for “lag” can be considered before the examined day to feed the data into the M-LSTM model to predict confirmed, death, and recovered cases. To find the optimum lag, data of all countries from 22 January 2020 till 30 July 2020 was used as the training set and the data from 1 August 2020 till 31 August2020 of a set of nine countries (Iran, China, Italy, Spain, Germany, Switzerland, Korea, Japan, and the USA) was used as test data.  Figure 4 is designed to show the MAPE values for predicting occurrences of confirmed, death, and recovered cases from COVID-19 when lags of 1-20 days are used on validation data in a preparatory model to find the optimum lag in the considered range. The lowest MAPE is found for lags of 6, 8, and 10 days; 5, 6, and 7 days; and 5, 6, and 18 days for confirmed, death, and recovered cases, correspondingly. Therefore, a lag of six days in all three cases is selected as the “optimal lag parameter.”

### 3.2. Optimal Model Selection

Five different models (Section 2.2) and three input settings (selected lag (previous occurrences) alone and adding basic and detailed features in the next two settings) are evaluated. A set of nine countries are selected for evaluation; China is undoubtedly the main candidate. Iran, Italy, Spain, and the USA are selected due to the report of a high number of confirmed and death cases. Germany and Switzerland are also coming from different trends with a high number of confirmed cases and a controlled number of deaths. Finally, Korea and Japan are also included in demonstrating the countries with a high degree of control on the epidemic. Tables 2, 3, and 4 show the performance of the model in the nine selected countries for the confirmed, death, and recovered groups. Concerning the results of Table 2, we found the best set of parameters, including basic and detailed features plus lag (previous occurrences). Furthermore, the results suggest that M-LSTM is the best performing network (winner model) for identifying the true magnitude of the pandemic with the best performance metrics: MAPE, RMSE, NRMSE, and *R*^2^ of 0.509%, 458.12, 0.001624, and 0.99997, respectively.  Figure 5 compares the ability of best- and worst-performing (RF) models in the correct prediction of the test values.

### 3.3. Future Trajectory of COVID-19 in Iran

As described above, data from all countries provided by John Hopkins University [28] from January 22 till July 30, 2020, was used as the training set. The test set is data from the nine mentioned countries between 1 August and 31 August 2020. Based on this test result in Tables 2, 3, and 4, the winner model (M-LSTM) is selected for forecasting the future trajectory of COVID-19 in Iran.

The forecasting results are illustrated in Figure 6. The predicted daily numbers of confirmed, death, and recovered cases in Iran are demonstrated in Figures 5(a)–5(c), respectively. We also show the cumulative numbers of all cases in Iran in Figure 5(d). To show the performance of the model in other countries mentioned, we also present the predictions by the proposed method in Appendix.

### 3.4. Effect of Country Actions on Predictions

In this paper, we propose a new scheme for modeling the “country actions” in Iran. Nationwide actions cannot be ignored during the modeling; however, the deep learning methods have no particular input indicating that. Accordingly, the trend of the time series in each time period is only dependent on actions made prior to that time point. To address this limitation, we stopped the training at different time points (each in accordance with distinct country actions). We expect that the predictions in each case confirm with prior actions, and any new action would result in a different curve. Therefore, if the action had a positive effect, the predicted number of infected people goes up compared to the real curve. On the other hand, the negative actions would lead to lower values in the predicted curve, indicating that a good scenario could happen without such incorrect actions. Three sample actions and occasions in Iran are considered in this paper:

- The nationwide closure of schools/universities, nonessential services, and public transportation in big cities before March 11, 2020
- Persian new year on March 19, 2020, and holiday trips (which was not banned officially and caused a great amount of transfer in Iran)
- Closure of roads between cities from March 27 to April 4, 2020

As shown in Figure 6, the training of the model (for prediction of confirmed cases) is stopped on three dates related to the occasions mentioned above. The blue curve on March 11 indicates that without first action, the curve could rise on March 11. On the other hand, the red curve shows a considerably lower peak could potentially happen if the second occasion would not happen. Finally, the green curve shows that the closure of roads would lead to a vanishing curve, which never happened due to the stop of this restriction and the following decisions.

## 4. Discussion

COVID-19 pneumonia started in late December 2019 and posed a continuing and dynamic threat globally. The first case was confirmed by February 19, 2020, in Iran. The main question of the public and politicians is the behavior of the epidemic, including the peak day, peak number, endpoint, and the daily number of new cases and deaths. Being aware of the real-time behavior of epidemics is vital for efficient logistics in the outbreak response. Forecast models will help the policymakers speculate the potential trajectory of the outbreaks and drive interventions as well as estimate the impact of interventions.

Five different models (Section 2.2) and three input settings (selected lag (previous occurrences) alone and adding basic and detailed features in the next two settings) are evaluated on a set of nine countries, and based on MAPE, RMSE, NRMSE, and *R*^2^ metrics, M-LSTM was the most accurate model found in this study. As mentioned before, it is not enough to only consider the information from one single day, so different time lags are considered before the examined day to feed the data into the model to predict confirmed, death, and recovered cases. This network uses lag information from confirmed, death, and recovered cases to predict the next occurrences. As an important issue, the number of days used as input and the output of prediction methods, the optimal lag of six days, and long-term (extendable to months) forecast are proposed in this study, unlike other studies that have a shorter forecast time [21, 22, 24, 26]. As shown in Table 2, all three groups (confirmed/death/recovered people) are used as the input of the selected model and to estimate one of the outputs. Therefore, the effect of all categories on the output is considered. This result shows that considering the mutual effect of these three occurrences can provide better modeling, and ignoring such dependence leads to less performance.

The basic assumption of the models is the stability of the environment measurements, but as we do not live in controlled conditions, every decision would change the epidemic track. As illustrated in Figure 6, by considering the stability of outbreak response, the first peak of the epidemic occurred around April 1st, with about 3000 new cases. The intersection of the predicted curve with observed data in Figures 6(a)–6(c) indicates the ability of correct forecasting by the proposed method.

Although the impact of actions of different countries on forecasts has been investigated in the articles, in this study, a new method was applied to investigate this effect on predictions. The training was stopped at different time points (each in accordance with distinct country actions). If actions of a country have a positive effect, the predicted number of infected people will increase compared to the actual curve; on the other hand, negative actions will lead to a decrease in the predicted curve values. The effect of governmental decisions and public occasions is illustrated in Figure 7. Considering that it takes around 5-6 days (the median of incubation period) for the results of interventions to show up on new case numbers, the difference between blue (predicted) and green (real effect of big closure in the country) curves between March 11 and 25 is the result of good decisions. However, the difference between red (predicted) and green (real effect of travels) between March 23 and April 2 is because of a bad occasion. By focusing on social distancing, there could be a steady decline in new cases after April 2 as shown by the green line, but changes in public health policies (like reopening of most public places in Iran or change in case of definition, testing availability, and the number of tests performed) reformulated the epidemic track, and the number of daily cases has started to go up as well.

Using this model, we aimed to identify (1) the intensity and the timing of the epidemic peak, (2) the total number of cases expected over the duration of the epidemic of COVID-19 in Iran, and (3) the effect of government policy on the number of infected cases. Determining these outcomes could improve resource allocation for risk communication, primary prevention, secondary prevention, and preparedness plans (e.g., planning medical staff and preparing triage units)

## 5. Conclusion

The recent outbreak of COVID-19 is affecting many countries worldwide including Iran as one of the top 10 most affected countries. In this study, we proposed the use of prediction models for COVID-19 incidence in Iran; our result could be useful in preparing for future outbreaks as well as the current one by considering the results in public health decision-making. Similar to other modeling techniques, the approach presented here is subject to limitations, which include data quality associated with real-time modeling (as data is often subject to ongoing cleaning, correction, and reclassification of onset dates as further data become available), reporting delays, and problems related to missing data. Predicting confirmed, death, and recovered cases can help healthcare organizations to identify logistical barriers related to medical equipment at the outbreak center and to rapidly build new local medical facilities. Furthermore, such predictions may help other countries that are now battling the outbreak to be more prepared. These measures are also essential to control the epidemic, protect frontline health workers, and reduce the severity of patient outcomes.

## Figures and Tables

**Figure 1:** The overall diagram of a RF.

**Figure 2:** The overall structure of the MLP network.

**Figure 3:** The overall structure of the LSTM model.

**Figure 4:** The MAPE values for predicting occurrences of confirmed, death, and recovered cases from COVID-19, when 1-20 days of lag are used in the preparatory model.

**Figure 5:** Comparison of the worst and the best performing models in the correct following of the training set and accurate prediction of the test values.

**Figure 6:** Forecasting (a) confirmed, (b) death, and (c) recovered daily values and performance of the forecasting after August 31 compared to real reported values and (d) cumulative values for Iran using the M-LSTM method.

**Figure 7:** Effect of country actions on predictions in Iran. The training on confirmed cases is stopped on three dates (dates March 11, March 23, and April 2 related to three sample decisions of the country). The deviation of curves from the real curve in the mentioned dates shows what could happen without such decisions.

**Figure 8:** Forecasting (a, e, i, m) confirmed, (b, f, j, n) death, and (c, g, k, o) recovered daily values and performance of the forecasting after August 31 compared to real reported values, and (d, h, l, p) cumulative values for Germany (first row), Italy (second row), Japan (third row), and Korea (fourth row) using the M-LSTM method.

**Figure 9:** Forecasting (a, e, i, m) confirmed, (b, f, j, n) death, and (c, g, k, o) recovered daily values and performance of the forecasting after August 31 compared to real reported values, and (d, h, l, p) cumulative values for Switzerland (first row), the USA (second row), Spain (third row), and China (fourth row) using the M-LSTM method.

**Table 1:** The best-selected architecture for each model and characteristics of each one.

Model	Layers	Filters
RF	*n* estimators = 300	Random state = 10
MLP	6	128, 128, 256, 256, 256, 1
LSTM-R	2 LSTM+2 dense	64, 32, 32, 1
LSTM-E	2 LSTM+2 dense	64, 32, 32, 1
M-LSTM	2 LSTM+2 dense	64, 32, 32, 1

**Table 2:** Comparison of performance in test stage on nine selected countries.

Model	BI	DI	Lag	MAPE	*R* ^2^ score	RMSE	NRMSE
RF			∗	2.34	0.99119	19497	0.069109
	∗		∗	2.6	0.98764	23103	0.081891
	∗	∗	∗	2.7	0.98741	23308	0.082617
MLP			∗	1.32	0.99422	499	0.001769
	∗		∗	1.7	0.99348	530	0.001879
	∗	∗	∗	1.54	0.99380	517	0.001833
LSTM-R			∗	2.260	0.98088	3242.91	0.011495
	∗		∗	2.032	0.98185	1065.41	0.003776
	∗	∗	∗	2.025	0.99023	1032.34	0.003659
LSTM-E			∗∗	1.213	0.99521	750.60	0.002661
	∗		∗∗	1.251	0.99671	610.86	0.002165
	∗	∗	∗∗	0.911	0.99832	580.41	0.002057
M-LSTM			∗∗	0.726	0.99884	530.74	0.001881
	∗		∗∗	0.550	0.99981	490.17	0.001737
	∗	∗	∗∗	**0.509**	**0.99997**	**458.12**	**0.001624**

∗ represents only confirmed cases as input and ∗∗ shows the confirmed cases along with death and recovered cases. BI: basic information; DI: detailed information. The performance is evaluated on **confirmed** cases as output.

**Table 3:** Comparison of performance in the test stage on nine selected countries.

Model	BI	DI	Lag	MAPE	*R* ^2^	RMSE	NRMSE
RF			∗	2.241	0.999988	111	0.00055
	∗		∗	3.996	0.999712	199	0.000986
	∗	∗	∗	11.852	0.998976	283	0.001402
MLP			∗	0.482	0.999991	20	0.000099
	∗		∗	1.320	0.999722	109	0.00054
	∗	∗	∗	0.990	0.999801	65	0.000322
LSTM-R			∗	1.549	0.999709	110.5	0.000547
	∗		∗	1.210	0.999799	107.4	0.000532
	∗	∗	∗	1.325	0.999714	109.2	0.000541
LSTM-E			∗∗	1.302	0.999790	108.1	0.000535
	∗		∗∗	1.112	0.999800	105.9	0.000524
	∗	∗	∗∗	0.960	0.999853	59.2	0.000293
M-LSTM			∗∗	0.641	0.999901	42.5	0.000210
	∗		∗∗	0.524	0.999956	31.9	0.000158
	∗	∗	∗∗	**0.481**	**0.999994**	**20.0**	**0.000099**

∗ represents only death cases as input and ∗∗ shows the confirmed cases along with death and recovered cases. BI: basic information; DI: detailed information. The performance is evaluated on **death** cases as output.

**Table 4:** Comparison of performance in test stage on nine selected countries.

Model	BI	DI	Lag	MAPE	*R* ^2^	RMSE	NRMSE
RF			∗	2.069	0.980306	2823	0.001057
	∗		∗	2.557	0.979987	3012	0.001128
	∗	∗	∗	2.580	0.979985	4620	0.00173
MLP			∗	0.337	0.999989	1059	0.000397
	∗		∗	1.686	0.980184	4634	0.001735
	∗	∗	∗	0.786	0.989893	3046	0.001141
LSTM-R			∗	2.030	0.980005	4963	0.0018658
	∗		∗	1.941	0.980102	4702	0.001761
	∗	∗	∗	1.536	0.986131	4369	0.001636
LSTM-E			∗∗	0.547	0.989981	1784	0.000668
	∗		∗∗	0.853	0.989634	2921	0.001093
	∗	∗	∗∗	0.624	0.989972	1991	0.000745
M-LSTM			∗∗	0.302	0.999991	1000	0.000374
	∗		∗∗	0.132	0.999997	621	0.000232
	∗	∗	∗∗	**0.073**	**0.999999**	**210**	**0.0000786**

∗ represents only recovered cases as input and ∗∗ shows the confirmed cases along with death and recovered cases. BI: basic information; DI: detailed information. The performance is evaluated on **recovered** cases as output.

**Table 5:** Comparison of performance in forecast stage on nine selected countries from September 1 to October 12.

Country	MAPE		
	Confirmed	Recovered	Deaths
Iran	0.45	0.19	0.79
Germany	0.778	0.27	1.01
Italy	1.2	0.84	0.81
Japan	1.22	0.41	0.98
Korea	0.71	1.31	1.1
Switzerland	0.64	0.43	0.47
The USA	0.23	0.75	0.35
Spain	0.95	0.7	0.01
China	0.21	1.75	0.96

## Data Availability

The data in this work is provided by John Hopkins University available in [28].

## Appendix

### Predictions on More Countries

Here, we present the predictions by the proposed model (M-LSTM and three input settings including basic and detailed features and lag) for Germany, Italy, Japan, and Korea in Figure 8 and for Switzerland, Spain, China, and the USA in Figure 9. As can be seen from the first to third columns in Figures 8 and 9, there is always a lag between the actual numbers and the predicted ones, but the model seems to work on a wide range of countries, which is encouraging. Also, a comparison of performance in the forecast stage from September 1 to October 12 on nine selected countries is summarized in Table 5.
